This article has been retracted.

# Case Management Improves Satisfaction, Anxiety, and Depression of Patients with Pregnancy Loss after In Vitro Fertilization and Embryo Transfer

**DOI:** 10.1155/2022/1968313

**Published:** 2022-04-07

**Authors:** Xiangli Wu, Yidan Wu, Mei Xia, Wenjie Xie, Huijing Hu, Zhen Xiao, Weihai Xu, Jing Shu

**Affiliations:** Center for Reproductive Medicine, Department of Reproductive Endocrinology, Zhejiang Provincial People's Hospital, Affiliated People's Hospital, Hangzhou Medical College, Hangzhou, 310014 Zhejiang Province, China

## Abstract

**Objective:**

Pregnancy loss has negative impacts on both the physical and the mental health of expectant mothers, which calls for an in-depth investigation. In this study, we examined the effects of case management on patients with pregnancy loss after in vitro fertilization and embryo transfer (IVF-ET).

**Methods:**

100 participants that had suffered pregnancy loss after IVF-ET-assisted pregnancy from January 2019 to March 2020 were divided into routine care and case management groups, each with 50 cases. For the routine care group, a doctor led the diagnostic and treatment processes and a nurse assisted with the treatment. For the case management group, a nurse led the patient diagnostic and treatment processes and a doctor controlled the diagnosis and treatment plan formulation. Case management models were established according to the comprehensive peripregnancy loss care of patients with pregnancy loss after IVF-ET-assisted pregnancy. The participants' outcomes (satisfaction, anxiety, and depression) were assessed at the time of pregnancy loss and 1 and 3 months after pregnancy loss during follow-up of the routine care and case management groups.

**Results:**

There was no statistical difference between the patients in the two groups with regard to their general information statistics (*P* > 0.05) or their satisfaction, anxiety, and depression at the time of pregnancy loss (*P* > 0.05). One month after pregnancy loss, there was no statistical difference in anxiety between the two groups (*P* > 0.05), but satisfaction was greater and depression was significantly reduced in the case management group compared with the routine care group (*P* < 0.05).

**Conclusion:**

Case management care can have a positive effect on improving the satisfaction, anxiety, and depression of patients that have had pregnancy loss after IVF-ET.

## 1. Background

Pregnancy and childbirth are highly significant experiences in a woman's life. Female infertility is diagnosed when a women has sex without contraception for at least 12 months but does not get pregnant [1]. There is no obvious difference in the incidences of infertility among regions; however, the incidence of infertility is increasing annually in China and has reached 10% to 15% [2]. In vitro fertilization and embryo transfer (IVF-ET) is an assisted reproductive technology that involves the fertilization of mature eggs with selected sperm in vitro, their development into embryos in a petri dish, and their implantation into the maternal uterine cavity for a normal pregnancy [3]. Since the birth of the world's first test-tube baby in 1978, IVF-ET has become the most effective way to treat infertility [4]. However, recent research has indicated that IVF-ET may cause 10%–50% of women to have symptoms of depression and anxiety [5]. The unpredictable results of IVF-ET may induce negative emotions, and patients often feel under stress while waiting for news of the outcome, during which time common reactions are anxiety and depression [6]. In addition, anxiety and depression in patients receiving IVF treatment may lead to a lower pregnancy rate [7–9]. Unfortunately, the pregnancy loss rate after IVF-ET remains high, and the live birth rate is approximately 20%–30%, which has become an important issue in assisted reproduction treatment [10]. Pregnancy loss, also called miscarriage or spontaneous abortion, is usually considered as the termination of pregnancy before 20 weeks of gestation [11], and the causes of pregnancy loss are complicated. The difficulty and uncertainty of diagnosis and treatment put patients and their families under tremendous pressure, which seriously affects their physical and mental health [12–16].

The nursing care of patients [17] after IVF-ET and pregnancy loss is an important service. However, routine nursing care based on a standardized diagnosis and treatment model can only ensure the presence of a nurse and the basic provision of treatment. Routine nursing care cannot provide holistic and continuous services for everyone [14]. To better serve patients, case management has been proposed, which is the coordinated implementation of health assessments, planning, care, and monitoring [18]. The case manager coordinates and integrates the opinions of various professionals to provide holistic and continuous care for the patient [17]. The concept of case management was first proposed in the United States as a patient-centered management method that focuses on coordinating, integrating, and providing medical care services, and it has been widely used in clinical practice [19–23]. In this model, the case manager is the spokesperson, manager, coordinator, counselor, and educator of patients and their families. Whether the application of case management can improve the physical and mental health of patients with pregnancy loss after IVF-ET is worth exploring.

This researcher explored the effects of case management on patients after IVF-ET pregnancy loss by comparing the general information, satisfaction, Self-Rating Anxiety Scale (SAS) score, and Self-Rating Depression Scale (SDS) score of patients in routine care and case management groups. This study provides information that can be used to help patients who have suffered pregnancy loss after IVF-ET to improve their satisfaction and alleviate their anxiety and depression.

## 2. Methods

### 2.1. Sampling and Data Collection

The participants were recruited from a reproductive medical center at a university hospital in the city of Hangzhou, the capital of and largest city in Zhejiang province on the east coast of China. Participants were referred through nurses of the clinic. Interviews were conducted in a quiet room of the outpatient clinic whenever it was convenient for the informants. There was no one else present during the interviews.

The participants were referred to the program with the following inclusion criteria: (a) participants that had suffered pregnancy loss after IVF-ET, (b) participants who had to undergo operative abortion, (c) participants who could communicate well and answer the investigators' questions independently, and (d) participants were willing to accept investigation and interventions. The exclusion criteria included participants who had a mental illness or were receiving medication and those who had had a recent major emergency in the family.

In this survey, a total of 121 questionnaires were distributed and 121 were recovered, with a response rate of 100%. There were 101 valid questionnaires and 20 invalid questionnaires that were incompletely filled by participants. One participant was excluded for marital reasons. Thus, a total of 100 participants were divided into routine care and case management groups, with 50 cases in each group.

### 2.2. Research Tool (Variables)

The following questionnaires were used in this study:

- General Information Questionnaire, which included age, education level, family monthly income, and pregnancy week
- Satisfaction Questionnaire, which included participants' attitude toward medical staff, waiting times, medical processes, and treatment results, with 5-grade evaluation standards (very dissatisfied, dissatisfied, fair, satisfied, and very satisfied). Cronbach's *α* was 0.86. The evaluation standards were given different scores using a 5-point Likert scale [11]. Generally, very dissatisfied equaled 1 point; dissatisfied, 2 points; general, 3 points; satisfied, 4 points; and very satisfied, 5 points
- Self-Rating Anxiety Scale (SAS) was developed by Zung [15] and measures the participant's self-evaluated anxiety. Cronbach's *α* was 0.82. This scale contains 20 items that reflect the patient's subjective feelings of anxiety. Each item is divided into four grades according to the frequency of symptoms, of which 15 are positive scores and 5 are negative scores. The participants conduct an independent self-assessment based on the actual situation in the past week without being influenced by others. The following scoring standards were used: none or very little of the time, a small amount of the time, a considerable amount of the time, and most or all the time. Each item was scored from 1 to 4 points. The total score of 20 items ranged from 20 to 80 points, and the standard score (25 to 100 points) was defined as the total score multiplied by 1.25. The cutoff value of the standard score was 50 points, and higher points represented higher anxiety
- Self-Rating Depression Scale (SDS) was developed by Zung and Gianturco in 1971 [16] and is mainly used to measure changes in patients' depression through self-assessment. Cronbach's *α* was 0.82. This scale contains 20 items that reflect the patient's subjective feelings of anxiety, and each item is divided into four grades according to the frequency of symptoms, of which 15 are positive scores and 5 are negative scores. The patient conducts an independent self-assessment based on the actual situation in the past week and is not affected by others. The following score standards were used: occasionally, sometimes, often, and continuously. Each item was scored from 1 to 4 points. The total score for the 20 items ranged from 20 to 80 points, and the standard score (25 to 100 points) was defined as the total score multiplied by 1.25. According to the Chinese standard, the cutoff value of the SDS standard score was 53 points, and 53 to 62 points represented mild depression; 63 to 72 points, moderate depression; more than 72 points, severe depression; and fewer than 53 points, normal. A higher score represented more severe depression

### 2.3. Interventions

The research team explained the study and interventions to the participants, including the time of outpatient clinic appointments; the purpose, duration, content, and significance of the research; and how to cooperate with the study. After obtaining informed consent, research tools were used to investigate the patients' situation. Routine care and case management services were assigned after the grouping.

#### 2.3.1. Routine Care Group

In the routine care group, the doctor led the process of diagnosis and treatment, and the nurse assisted in the treatment. Specifically, the participants went to the outpatient clinic, and the receiving doctor diagnosed and analyzed their condition. Those who needed to undergo abortion went through a preoperative examination, preoperative discussion, and consent submittal. The outpatient nurse then explained to each patient the purpose, time, content, and significance of the study and how to cooperate. After obtaining their informed consent, the nurse used research tools to investigate the basic medical conditions of the participants. The operating room nurse was responsible for the abortion operation arrangements. Before abortion, periabortion education was conducted, preoperative inspection was performed, and preoperative precautions were presented. In the intraoperative period, doctors provided a safe and relaxing environment for the participants. In the postoperative period, the participants were transported safely and vital signs were observed. The doctor then explained the medication, follow-up time, and other precautions taken after abortion. The participants underwent the treatment according to routine procedures provided by the doctor. Afterwards, the nurse used research tools to investigate the participant's health 1 month and 3 months after abortion.

#### 2.3.2. Case Management Group

In the case management group, the nurse led the diagnosis and treatment processes and the receiving doctor was responsible for the participants' diagnosis and treatment plan formulation. A platform for communication between medical staff and the participants and their families regarding pregnancy loss investigation and case management models, such as education and psychosocial support for reproductive health, was established according to the comprehensive peripregnancy loss care of patients with pregnancy loss after IVF-ET-assisted pregnancy.

The following steps were taken to evaluate the case management group. First, the case manager introduced him-/herself and explained the purpose, duration, content, and significance of the study and how to cooperate. After obtaining informed consent, research tools were used to investigate the participant's basic situation, and a case management file that included detailed records of the participant's basic information and medical history was established. The case manager exchanged contact information, such as telephone number and WeChat information, with the participants. Participants were encouraged to join a “pregnancy loss mutual aid group,” via which the case manager could dynamically track and educate the patients and judge the development of their condition in real time; using this information, the case manager could provide feedback on the participant's condition to the attending doctor and participate in discussions with the medical team.

The following steps were involved in intervention planning. The case manager conducted a comprehensive analysis of the information obtained during the evaluation, the participant's actual situation, and the expected goals and arranged for the participants to be seen by a reproduction specialist. The doctor diagnosed and treated the participants and determined the cause of pregnancy loss or performed other related examinations. The most appropriate treatment plan and goals according to patient type were then formulated. The plan was clinically centered and based on individual patient information.

The next stage of the intervention was the implementation of care. Based on the results of the questionnaire, the case manager assessed the participant's family and social relationships and gave the patient appropriate psychological interventions based on the actual situation, organized her treatment and medical procedures, and accelerated the patient's adaptation to the hospital environment, which included encouraging the participants to indulge in appropriate distractions (such as reading and other entertainment) to prevent them from focusing on their situation, reduce their emotional responses to stress, and enhance their confidence in fighting the condition. The use of online platforms to establish good nurse–patient relationships with participants and their families based on respect and trust was also encouraged. The case manager then provided pregnancy-loss-related education in the “pregnancy loss mutual aid group” and distributed educational materials on pregnancy loss to the participants and information on how provide support to their spouse and family. In addition to the conventional peripregnancy period and pregnancy loss education content, the case management division provided preoperative education to the participants, as well as embryonic villus chromosome detection and/or other specific examinations that have significance in the analysis of the cause of pregnancy loss and the success of the next pregnancy. In the postoperative period, the case manager gave the patients relevant medical guidance according to the doctor's orders and guided the postoperative precautions, including medication status, recent contraceptive methods, and contraceptive and follow-up times. During this period, telephone interventions and education by case managers were accepted. Postoperative follow-up was performed three times:

The first follow-up was conducted by telephone or online platform in the first week after abortion, during which the patients were asked about their physical condition, including blood loss volume and whether there was abdominal pain or not. The researchers gathered information on the patients' living habits, husbands' attitude, family's attitude, living environment, and family support. If there were any particular needs or issues raised, feedback was quickly given to the doctor, who passed information on to the psychologist about poor psychological scale scores. The psychiatrist formulated a treatment plan for the patient based on their opinions and communicated with the doctor for no less than 20 minutes each time. The second follow-up occurred when the results of the villi gene test were obtained in the second week after abortion, at which point the researchers contacted the participants by the network platform or telephone. Then, appropriate explanations were made according to the results, and the participants were booked for a review 1 month after abortion. The researchers also discussed the doctor's advice with the patient. Each communication lasted at least 20 minutes.

The third follow-up was 4-5 weeks after the abortion. The case manager arranged a doctor to visit the patient for an examination, questioned patients about their medical needs and problems with psychological adjustment at any time during the period, encouraged the support provided by family members, and encouraged two-way feedback. Each communication lasted for no less than 20 minutes, and the case manager conducted a second patient questionnaire. During the intervention period, clear lines of communication were of the utmost importance, and the case management model was applied to the whole process of nursing care, allowing timely evaluation of the mental health of patients and their satisfaction with the medical services and treatment outcomes.

Next, the case manager attended to the participants' examination results from the IVF-ET-assisted pregnancy period and comprehensive follow-up results, rapidly and correctly judged the development of the condition, provided timely feedback to the attending doctor, participated in discussions with the medical team, and notified the participants and family of the final diagnosis, treatment opinions, and suggestions made by the medical team.

The last step was monitoring. The case manager used the research tools to investigate the participants' condition 1 and 3 months after pregnancy loss. During the treatment, the case manager monitored the patient's postabortion conditions, including bleeding, infection, uterine adhesions, and endometrial repair, and communicated with the attending doctor to discuss treatment plans. Any problems with service implementation were recorded, so they can be analyzed and improved.

### 2.4. Statistical Analysis

The questionnaires completed by the participants were retrieved on the spot by the members of the research team and checked for validity and completeness. The data were entered into a database after double-checking their validity. SAS 9.4 software was used for statistical analysis. Categorical variables were expressed in the form of frequency (percentage), and the chi-square test was used to compare the group statistics. As the quantitative data did not conform to a normal distribution, the median (and lower and upper quartiles) was used in the descriptions. The rank sum test was used for comparisons between groups.

## 3. Results

### 3.1. General Participant Information

The general information on the participants, including age, educational level, occupation, family monthly income, payment status, and gestational age, showed no statistical difference between the two groups (*P* > 0.05) (Table 1).

### 3.2. Comparison of Satisfaction between Patients in the Two Groups

Table 2 shows there was no significant difference between the two groups' satisfaction scores at the time of pregnancy loss (*P* > 0.05), while Table 3 shows that the satisfaction of the case management group was higher than that of the routine care group at 1 month after pregnancy loss (*P* < 0.05).

### 3.3. Comparison of Anxiety and Depression of Participants in Two Groups at Pregnancy Loss

As demonstrated in Table 4, the survey showed no significant differences in anxiety and depression between the two groups at the time of pregnancy loss (*P* > 0.05), while at 1 month after pregnancy loss, depression was lower in the case management group than in the routine care group, and the difference was statistically significant (*P* < 0.05) (Table 5). However, there was no significant difference in anxiety between the two groups 1 month after pregnancy loss (*P* > 0.05).

## 4. Discussion

IVF-ET is the most effective way to treat infertility; however, pregnancy loss after IVF-ET is still high, and IVF-ET may cause participants to feel depressed and pressured [24, 25]. In this study, we explored the effects of case management on participants with pregnancy loss after IVF-ET. Compared with the routine care group, the case management group showed improvements in their satisfaction and depressive emotions.

IVF-ET is currently one of the most important and effective methods used for treating infertility [26]. According to a recent study, participants expressed dissatisfaction after pregnancy loss following IVF-ET, which is consistent with previous studies showing that participants with pregnancy loss were likely to express dissatisfaction [27, 28]. However, few studies have reported on the application of case management for participants who have had pregnancy loss after IVF-ET [29]. Here, we showed that, at the time of pregnancy loss, participants who suffered pregnancy loss after IVF-ET and were provided case management were equally as satisfied as pregnancy loss patients given routine care, whereas 1 month after the pregnancy loss, participants in the case management group had a higher level of satisfaction than those in the routine care group. Therefore, we suggest that case management can respond to the needs of participants effectively and improve participants' satisfaction with all aspects of hospital care. The potential benefits of case management were put forward several years ago, and case management has been applied in numerous medical fields, including those of tumor [30], coronary disease [31], HIV [32], Alzheimer's disease [33], and low-weight children [34]. Park et al. [35] proposed using case management to improve participants' satisfaction, mainly involving individualized treatment, the attention of case managers, and emotional support.

Pregnancy loss is a psychological stressor and increases the patient's mental health burden [36], and anxiety and depression are the main results of pregnancy loss after IVF-ET [37]. Cui et al. [38] reported that depression has a negative impact on pregnancy outcomes following IVF-ET. Compared with naturally conceiving women, women who received IVF treatment had more severe anxiety symptoms and higher levels of stress biomarkers [39]. Our findings are consistent with these previous results and showed that participants who had pregnancy loss after IVF-ET were more likely to feel anxious and depressed. Therefore, it is important to help people with pregnancy loss after IVF-ET to prevent anxiety and depression. Case management has been reported to be useful as a high-risk prenatal care strategy, providing individualized management for complex cases and facilitating the flow of information between health services, concreting the comprehensiveness and quality of the care [40]. The Anxiety and Depression Scale was used to measure participants' mental health. Analysis showed that SAS scores were not significantly different between routine care and case management groups, the reason being that, generally, participants who suffered pregnancy loss after IVF-ET experienced many other difficulties, such as long bleeding times, fetal care issues, an abnormal uterus or fetus, long-term undiagnosed miscarriages, and urgent reproductive requirements, which increase the complexity of pregnancy loss [41]. However, this study found the SDS scores of participants in the case management group to be significantly lower than those in the routine group 1 month after pregnancy loss, indicating that case management can help relieve depression in participants. Similar to our findings, case management has been reported to help relieve anxiety in participants with depressive and anxiety disorders [42]. Taube et al. [43] found that case management can relieve the symptom of depression in community-dwelling older people, and Ogburn et al. [32] reported that case management services had a positive effect on the success of depression treatment, all of which support the idea that case management can provide benefits in clinical nursing care and health guidance for people that have experienced pregnancy loss after IVF-ET-assisted pregnancy.

This study found that case management improves the physical and mental health of these patients, and we encourage the in-depth development of reproductive health medical services with a certain degree of innovation. However, due to time restraints and other objective factors, the number of samples was not sufficient. Moreover, other relevant factors that may have led to deviations in some results were not analyzed. Investigations with larger samples should be continued in the future to improve the reliability of the research results and provide more information and practical guidance for clinical nursing.

## 5. Conclusion

This study examined the anxiety, depression, and satisfaction of Chinese couples during medical care after pregnancy loss following IVF-ET. These findings provide insights into the need to provide particular attention to patients after pregnancy loss following IVF-ET and point to a need for case management plans for these individuals.

## Figures and Tables

**Table 1:** Comparison of general information between the patients in the two groups.

Category	Routine care group	Case management group	*T* value/*χ*^2^ value	*P* value
Age	32.73 ± 5.42	31.33 ± 4.74	1.23^∗^	0.22
Education(%)			1.01^#^	0.32
Primary school or below	3 (6%)	4 (8%)		
Junior	18 (36%)	20 (40%)		
College degree or above	29 (58%)	26 (52%)		
Family monthly income (%)			-0.15^#^	0.88
<6000	9 (18%)	10 (20%)		
6000-8999	26 (52%)	25 (50%)		
9000-11999	3 (6%)	2 (4%)		
12000-15000	4 (8%)	3 (6%)		
>15000	8 (16%)	9 (18%)		
Gestational weeks	8.53 ± 1.68	8.60 ± 1.96	0.18^∗^	0.86

^∗^ *T* value, ^#^*χ*^2^ value.

**Table 2:** Comparison of satisfaction scores between the two groups of patients at the time of pregnancy loss [median (lower quartile, upper quartile)].

Satisfaction project	Routine care group (*n* = 50)	Case management group (*n* = 50)	*χ* ^2^ score	*P* score
Satisfaction with service attitude of medical staff	8 (8,10)	8 (8,10)	0.01	0.92
Satisfaction with waiting time	19 (17,20)	19 (17,20)	0.05	0.83
Satisfaction with the medical process	32 (31,35.5)	32 (31,35.5)	0.00	1.00
Satisfaction with treatment results	12 (11,12)	12 (11,12)	0.05	0.83

**Table 3:** Comparison of satisfaction scores between the two groups of patients one month after pregnancy loss [median (lower quartile, upper quartile)].

Satisfaction project	Routine care group	Case management group	*χ* ^2^ score	*P* score
	(*n* = 50)	(*n* = 50)		
Satisfaction with service attitude of medical staff	8 (8,10)	10 (10,10)	24.47	0.001
Satisfaction with waiting time	19 (17,20)	22 (20,24)	26.59	0.001
Satisfaction with the medical process	32 (31,35.5)	38.5 (34.5,40)	21.80	0.001
Satisfaction with treatment results	12 (11,12)	14 (13,15)	31.32	0.001

**Table 4:** Comparison of anxiety (SAS) and depression (SDS) scores in the two groups of patients at the time of pregnancy loss.

Group	Number	SAS score	SDS score
Routine care group	50	51.95 ± 8.32	60.65 ± 5.05
Case management group	50	51.40 ± 6.45	59.08 ± 6.30
*T* score		0.33	0.67
*P* score		0.742	0.507

**Table 5:** Comparison of anxiety (SAS) and depression (SDS) scores between the two groups of patients at one month after pregnancy loss.

Group	Number	SAS score	SDS score
Routine care group	50	50.63 ± 6.18	58.85 ± 5.90
Case management group	50	49.08 ± 6.36	55.28 ± 4.12
*T* score		-1.11	-3.14
*P* score		0.27	0.01

## Data Availability

The data used to support the findings of this study are available from the corresponding authors upon reasonable request.

## Additional Points

*Highlights*. (1) The satisfaction score in the case management group was statistically significantly higher than that of the routine care group. (2) The SDS score in the case management group was statistically significantly lower than that of the routine care group. (3) The SAS score in the case management group was lower than that of the routine care group.

## References

[1] Inhorn M. C., Patrizio P. (2015). Infertility around the globe: new thinking on gender, reproductive technologies and global movements in the 21st century. *Human Reproduction Update*.

[2] Karimzadeh M., Salsabili N., Akbari Asbagh F., Teymouri R., Pourmand G., Soleimanieh Naeini T. (2017). Psychological disorders among Iranian infertile couples undergoing assisted reproductive technology (ART). *Iranian Journal of Public Health*.

[3] Wang X., Wang W., Qu Q., Zhang N., Hao C., Ma D. (2019). Effect of large follicle puncture on IVF-ET outcome in patients with unsynchronized follicle maturationcan. *The Journal of International Medical Research*.

[4] Luo L., Fan X. Z., Jie H. Y. (2019). Is it worth reducing twins to singletons after IVF-ET? A retrospective cohort study using propensity score matching. *Acta Obstetricia et Gynecologica Scandinavica*.

[5] Namdar A., Naghizadeh M. M., Zamani M., Yaghmaei F., Sameni M. H. (2017). Quality of life and general health of infertile women. *Health and Quality of Life Outcomes*.

[6] Nicoloro-SantaBarbara J., Busso C., Moyer A., Lobel M. (2018). Just relax and you'll get pregnant? Meta-analysis examining women's emotional distress and the outcome of assisted reproductive technology. *Social Science & Medicine*.

[7] Gameiro S., Boivin J., Dancet E. (2016). Qualitative research in the ESHRE guideline 'routine psychosocial care in infertility and medically assisted reproduction - a guide for staff'. *Human Reproduction*.

[8] Li X. H., Ma Y. G., Geng L. H., Qin L., Hu H., Li S. W. (2011). Baseline psychological stress and ovarian norepinephrine levels negatively affect the outcome of in vitro fertilisation. *Gynecological Endocrinology*.

[9] Turner K., Reynolds-May M. F., Zitek E. M., Tisdale R. L., Carlisle A. B., Westphal L. M. (2013). Stress and anxiety scores in first and repeat IVF cycles: a pilot study. *PLoS One*.

[10] Eroglu S., Colak E., Erinanc O. H. (2020). Serum and placental periostin levels in women with early pregnancy loss. *Journal of Reproductive Immunology*.

[11] Kim C. E., Shin J. S., Lee J. (2017). Quality of medical service, patient satisfaction and loyalty with a focus on interpersonal-based medical service encounters and treatment effectiveness: a cross-sectional multicenter study of complementary and alternative medicine (CAM) hospitals. *BMC Complementary and Alternative Medicine*.

[12] Kim G. S., Ko I. S., Lee T., Kim E. J. (2014). Effects of community-based case management by visiting nurses for low-income patients with hypertension in South Korea. *Japan Journal of Nursing Science*.

[13] Mills T. A., Ricklesford C., Cooke A., Heazell A. E., Whitworth M., Lavender T. (2014). Parents’ experiences and expectations of care in pregnancy after stillbirth or neonatal death: a metasynthesis. *BJOG*.

[14] Park C. S., Park E. (2018). Factors influencing patient-perceived satisfaction with community-based case management services. *Western Journal of Nursing Research*.

[15] Zung W. W. (1971). A rating instrument for anxiety disorders. *Psychosomatics*.

[16] Zung W. W., Gianturco J. A. (1971). Personality dimension and the self-rating depression scale. *Journal of Clinical Psychology*.

[17] White C. W., Alejandro J. (2020). Highly reliable case management. *Professional Case Management*.

[18] Fraser K. (2020). Case management. *Professional Case Management*.

[19] Dieterich M., Irving C. B., Bergman H. (2017). Intensive case management for severe mental illness. *Cochrane Database of Systematic Reviews*.

[20] Joo J. Y., Liu M. F. (2018). Experiences of case management with chronic illnesses: a qualitative systematic review. *International Nursing Review*.

[21] King A. J. L., Johnson R., Cramer H., Purdy S., Huntley A. L. (2018). Community case management and unplanned hospital admissions in patients with heart failure: a systematic review and qualitative evidence synthesis. *Journal of Advanced Nursing*.

[22] Tsai C. Y., Li I. C., Lai F. C. (2018). Substantial effects of empowerment case management on physical health of type 2 diabetic patients. *Journal of Clinical Nursing*.

[23] van Eeden A. E., van de Poll I., van Vulpen G. (2017). Effectiveness of case management in the prevention of COPD re-admissions: a pilot study. *BMC Research Notes*.

[24] Egerup P., Kolte A. M., Larsen E. C., Krog M., Nielsen H. S., Christiansen O. B. (2016). Recurrent pregnancy loss: what is the impact of consecutive versus non-consecutive losses?. *Human Reproduction*.

[25] Joo J. Y., Huber D. L. (2014). An integrative review of nurse-led community-based case management effectiveness. *International Nursing Review*.

[26] Zhong Y., Li J., Ying Y. (2012). The efficacy of conversion from IUI to IVF-ET in infertility patients with hyper-response to ovulation induction: a retrospective study. *Biomedical Papers of the Medical Faculty of the University Palacky, Olomouc, Czech Republic*.

[27] He L., Wang T., Xu H. (2019). Prevalence of depression and anxiety in women with recurrent pregnancy loss and the associated risk factors. *Archives of Gynecology and Obstetrics*.

[28] Kolte A. M., Olsen L. R., Christiansen O. B., Schmidt L., Nielsen H. S. (2019). Pregnancy outcomes after recurrent pregnancy loss: a longitudinal cohort study on stress and depression. *Reproductive Biomedicine Online*.

[29] Yang J. H., Yang P. K., Chen M. J., Chen S. U., Yang Y. S. (2017). Management of endometrial polyps incidentally diagnosed during IVF: a case-control study. *Reproductive Biomedicine Online*.

[30] Scherz N., Bachmann-Mettler I., Chmiel C. (2017). Case management to increase quality of life after cancer treatment: a randomized controlled trial. *BMC Cancer*.

[31] Allen J. K., Blumenthal R. S., Margolis S., Young D. R., Miller E. R., Kelly K. (2002). Nurse case management of hypercholesterolemia in patients with coronary heart disease: results of a randomized clinical trial. *American Heart Journal*.

[32] Ogburn D. F., Schoenbach V. J., Edmonds A. (2019). Depression, ART adherence, and receipt of case management services by adults with HIV in North Carolina, Medical Monitoring Project, 2009-2013. *AIDS and Behavior*.

[33] Doty L., Heilman K. M., Stewart J. T., Bowers D., Rothi L. J. (1993). Case management in Alzheimer's disease. *Journal of Case Management*.

[34] Nyishime M., Borg R., Ingabire W. (2018). A retrospective study of neonatal case management and outcomes in rural Rwanda post implementation of a national neonatal care package for sick and small infants. *BMC Pediatrics*.

[35] Park C. S., Yoon S. L., Yun S. N., Park E. (2017). Korean patient-perceived satisfaction scale of community-based case management services (Korean-PSCCM): development and psychometric evaluation. *Journal of Community Health Nursing*.

[36] Zhang Y. X., Zhang X. Q., Wang Q. R. (2016). Psychological burden, sexual satisfaction and erectile function in men whose partners experience recurrent pregnancy loss in China: a cross-sectional study. *Reproductive Health*.

[37] Lang J., Zhang B., Meng Y., Du Y., Cui L., Li W. (2019). First trimester depression and/or anxiety disorders increase the risk of low birthweight in IVF offspring: a prospective cohort study. *Reproductive Biomedicine Online*.

[38] Cui Y., Yu H., Meng F., Liu J., Yang F. (2020). Prospective study of pregnancy outcome between perceived stress and stress-related hormones. *The Journal of Obstetrics and Gynaecology Research*.

[39] Garcia-Blanco A., Diago V., Hervas D., Ghosn F., Vento M., Chafer-Pericas C. (2018). Anxiety and depressive symptoms, and stress biomarkers in pregnant women after in vitro fertilization: a prospective cohort study. *Human Reproduction*.

[40] Soares L. G., Higarashi I. H. (2019). Case management as a high-risk prenatal care strategy. *Revista Brasileira de Enfermagem*.

[41] Bates G. W., Ginsburg E. S. (2002). Early pregnancy loss in in vitro fertilization (IVF) is a positive predictor of subsequent IVF success. *Fertility and Sterility*.

[42] Kivelitz L., Schulz H., Melchior H., Watzke B. (2015). Effectiveness of case management-based aftercare coordination by phone for patients with depressive and anxiety disorders: study protocol for a randomized controlled trial. *BMC Psychiatry*.

[43] Taube E., Kristensson J., Midlov P., Jakobsson U. (2018). The use of case management for community-dwelling older people: the effects on loneliness, symptoms of depression and life satisfaction in a randomised controlled trial. *Scandinavian Journal of Caring Sciences*.

